The article "Impact of Optimizing the Emergency Care Process on the Emergency Effect and Prognosis of Patients with Hepatic Encephalopathy" was published in 2022. Journal: Emerg Med Int.

# Impact of Optimizing the Emergency Care Process on the Emergency Effect and Prognosis of Patients with Hepatic Encephalopathy

**DOI:** 10.1155/2022/4446215

**Published:** 2022-08-24

**Authors:** Fang Wei, Haihong Tan, Yubiao He, Xin Shu

**Affiliations:** Department of Infection, Xiangya Second Hospital, Central South University, Changsha, Hunan Province 410011, China

## Abstract

Hepatic encephalopathy (HE) is a serious complication caused by liver disease and is one of the leading causes of death in patients. Studies have shown that proper emergency care for patients after the occurrence of HE can improve their prognosis and quality of life. Therefore, this study focuses on the effect of optimizing the emergency care process on the effectiveness and prognosis of emergency care for patients with hepatic encephalopathy. In this study, we set 32 patients with HE admitted to receive routine emergency care between May 2020 and March 2021 as the control group and 34 patients with HE admitted to receive optimized emergency care processes between April 2021 and February 2022 as the observation group. The satisfaction of patients' families with this care was assessed using a self-administered nursing satisfaction questionnaire to record the outcome of emergency care, quality of care, and prognosis of patients in the two groups of palliative care. The data collected were analyzed using SPSS17.0 software, and the results showed that the time spent on diagnosis, resuscitation, DTP, and DTT was much lower in the observation group than in the control group, and the scores related to the quality of care, such as ambulance technique, humanistic care, resuscitation efficiency, and resuscitation effect, were all higher than those of the control group, and the satisfaction of the family members in the observation group was also significantly higher than that of the control group (*P* < 0.05). The success rate of first aid in the observation group was 100.00%, which was higher than 93.72% in the control group, but the difference between the two groups was not significant (*P* > 0.05). It can be seen that the application of an optimized emergency nursing process in HE patients is effective, which can effectively improve the success rate of HE resuscitation, shorten the resuscitation time and condition diagnosis, improve the resuscitation effect, improve the quality of nursing care, and improve the prognosis of patients to a certain extent.

## 1. Introduction

Hepatic encephalopathy (HE) is a potentially serious complication occurring in patients with acute and chronic states, which can occur in 60–80% of cirrhotic patients and is clinically characterized by a complex array of nonspecific neurological and psychiatric symptoms [1, 2]. Because it often starts insidiously, most patients do not seek treatment until the late stage of the disease, when they are mostly in critical condition with complex changes, and if emergency care is not timely or inappropriate, it may affect the quality of life of patients in the later stages, and in serious cases, it may be life-threatening [3, 4]. Due to the complex and diverse pathophysiological basis of HE, the pathogenesis of HE has not been fully elucidated yet, and the theory of ammonia toxicity is still the core of the theory that high blood ammonia is one of the main causes of HE [5, 6]. Regarding the treatment of HE, some studies [7] have pointed out that early identification of predisposing factors for the occurrence of HE and targeted indicators are key and that lactulose is the drug of choice for the treatment of recurrent HE, while rifaximin is considered an effective complementary treatment for the prevention of HE recurrence.

The article "Impact of Optimizing the Emergency Care Process on the Emergency Effect and Prognosis of Patients with Hepatic Encephalopathy" was published in 2022. Journal: Emerg Med Int.

Studies [8, 9] have shown that standardized and procedural emergency procedures are crucial in the treatment of HE, and emergency care is a holistic and comprehensive nursing intervention in the process of resuscitation of patients, which can effectively improve the success rate of resuscitation and facilitate the recovery of patients' conditions. However, there is a lack of unified standards and norms regarding the systematic nursing process, and there are many participants with the unclear division of responsibilities and division of labor, which can easily lead to a busy, disorganized, and inefficient resuscitation process [10]. It not only causes waste of manpower and time but also delays the resuscitation time and causes medical disputes. In recent years, along with the increase in the incidence of HE in China, the optimized nursing emergency process meets the current development of emergency department nursing as well as the actual clinical needs [11, 12]. This study compares the effect of 66 cases admitted to our hospital from May 2020 to February 2022 on the treatment of HE patients given conventional nursing emergency procedures and optimized nursing emergency procedures, respectively, and is reported below.

## 2. Information and Methods

### 2.1. Research Data

#### 2.1.1. Subjects and Grouping

66 HE patients admitted to our hospital from May 2020 to February 2022 were selected for this study, and the patients were divided into a control group (33 cases: conventional nursing emergency process, admitted from May 2020 to March 2021) and an observation group (34 cases: optimized nursing emergency process, admitted from April 2021 to February 2022) according to the order of admission.

The article "Impact of Optimizing the Emergency Care Process on the Emergency Effect and Prognosis of Patients with Hepatic Encephalopathy" was published in 2022. Journal: Emerg Med Int.

#### 2.1.2. Inclusion Criteria

Inclusion criteria were defined as follows: (1) history of severe liver disease and/or extensive portal-body shunt, neuropsychiatric symptoms, and signs, all confirmed by CT examination, evoked potential examination, and blood ammonia test; (2) informed consent has been obtained from the patient or family for all treatments and tests; and (3) admission within 2 to 48 h after the appearance of HE.

#### 2.1.3. Exclusion Criteria

Exclusion criteria were defined as follows: (1) patients who have received other treatments prior to admission to the hospital for emergency care; (2) suffering from severe immune system or hematologic disorders or other serious organ dysfunction; (3) suffering from malignant tumors; (4) having a history of psychosis or psychiatric disorders; (5) no other disabling or fatal diseases of the head; and (6) other diseases that might cause neuropsychiatric abnormalities, such as psychiatric diseases, toxic encephalopathy, intracranial lesions, other metabolic encephalopathies, and sedative overdose.

### 2.2. Study Methods

#### 2.2.1. Data Collection

The clinical data of patients who met the criteria, including gender, age, place of residence, smoking history, drinking history, underlying diseases, etiology, and causative factors, were recorded in detail by reviewing medical records on a copy-by-copy basis to establish a database.

#### 2.2.2. Control Group

Routine emergency nursing procedures were performed:

1. General emergency measures: after the emergency department staff received the patient, they assessed whether the patient had personality and behavior changes, abnormal consciousness, coma, jaundice, fluttering wing-like tremor, etc. The nursing staff prepared all kinds of resuscitation items such as suction materials, infusion materials, emergency care, cardiac monitor, restraint belt, enema materials, etc., and kept calm and collected throughout the whole process to quickly and skillfully cooperate with the resuscitation. By determining the patient's consciousness and circulation of the limbs, the patient was assisted to assume a flat position with the pillow removed, the patient's limbs were restrained, the patient's pupils were checked, and the physician was notified for resuscitation. Cardiac monitoring was given, intravenous access was established, and resuscitation measures such as blood transfusion, fluid transfusion, anti-infection, various hemostatic treatments, and medications were implemented in cooperation with the physician after emergency assessment of the patient's condition, and treatment effects and adverse reactions were observed. For some conscious patients, certain encouragement and comfort were given to increase patients' belief in survival.
2. After the condition was stabilized, closely observe the patient's vital signs, major symptoms, and physical signs, and immediately inform the doctor of any abnormalities and cooperate with the treatment.
3. Nursing staff reassessed the patient's physical condition and severity of illness, applied antihepatic encephalopathy drugs, actively treated the primary disease, and corrected metabolic disorders and water and electrolyte disorders in a timely manner according to medical advice. They promptly explained the condition to the patient's family, did a good job of psychological guidance for the family, eliminated all unsafe factors in the ward, and transferred the patient to a safe bed to avoid accidents. When the patient appeared irritable, do not abuse sedatives to avoid aggravating hepatic coma, and use a restraint belt if necessary.

The article "Impact of Optimizing the Emergency Care Process on the Emergency Effect and Prognosis of Patients with Hepatic Encephalopathy" was published in 2022. Journal: Emerg Med Int.

#### 2.2.3. Observation Group

Optimized emergency flow nursing was performed, with the following specific contents:

1. Optimize the consultation process: before the patient was admitted to the hospital, the emergency department nurse informed the ward to prepare for the admission of the patient, and the responsible nurse sent the patient directly to the resuscitation room after receiving the patient and completed the assessment of the patient's condition within 2 min, following the principle of “one look, two questions, three checks” to determine whether the patient had any fatal risk factors. Blood pressure, pulse rate, oxygen saturation, and consciousness were assessed every 15 minutes.
2. Optimize the ambulance process: ① implement prehospital-in-hospital integrated ambulance, before the ambulance arrives, telephone the family to instruct the awake patient to adopt a flat position, and if possible, give oxygen and remove respiratory secretions to avoid obstruction of the respiratory tract by vomit or resuscitation. ② open the green channel, and one prescreening nurse informed the internist and assisted the family to register, and another one immediately prepared various resuscitation items to cooperate with the resuscitation. ③ establishment of emergency field auxiliary center, by the unified training of field personnel to send specimens, transport patients, etc., to save time in all aspects and improve the efficiency of treatment. ④ establish intravenous access; the patient's condition is complicated and changeable in the process of resuscitation, and multiple drugs need to be used constantly for treatment, so more than two intravenous accesses should be established in time to facilitate infusion and timely injection of resuscitation drugs. ⑤ Re-evaluate the patient's physical condition and severity of illness, and observe the patient's vital signs, including blood pressure, pulse rate, and finger pulse oxygen saturation every 10–15 min, paying attention to the patient's temperature change and systemic response.
3. The emergency department holds monthly departmental meetings to summarize the problems in emergency department nursing as the first witness to HE treatment, and in order to improve the level of emergency nursing staff, HE-related emergency nursing skills training should be conducted regularly, while paying attention to the impact caused by the patient's family during the patient's emergency and timely reassuring the patient's emotions.

The article "Impact of Optimizing the Emergency Care Process on the Emergency Effect and Prognosis of Patients with Hepatic Encephalopathy" was published in 2022. Journal: Emerg Med Int.

### 2.3. Observed Indicators

(1) Effectiveness of first aid: assessed according to the time indicators of each part of the process, including the time from admission to seeing the emergency physician (door to physician, DTP), the time from admission to the emergency team (door to stoke team, DTT), the resuscitation time, and the diagnosis time of the condition. (2) Clinical outcome indicators: the clinical outcomes of cured discharge, improved discharge, and death were recorded for both groups. (3) Quality of nursing care: the quality of nursing care assessment scale was developed with reference to relevant literature, including four items of ambulance technique, humanistic care, resuscitation efficiency, and resuscitation effect, with a total score of 10 for each item. (4) Family satisfaction: the families of patients in both groups evaluated the degree of satisfaction with clinical care based on the dimensions of emergency speed, professionalism of the emergency nursing staff, and sense of responsibility for emergency care, with a score interval of 10 points for each item and a total score of 30 points, 30 being very satisfied, 15–29 being basically satisfied, and less than 14 being unsatisfied, with satisfaction = ((very satisfied + basically satisfied)/total number of cases) × 100%.

### 2.4. Statistical Methods

SPSS21.0 was applied to process the variable data, *n* (%) was used to express the relevant count data, and the *χ*^2^ test was used to express the relevant measurement data. The measurement data were described by means ± standard deviation (mean ± SD), and independent samples *t*-test was performed to compare the two groups. *P* < 0.05 indicates that the differences between groups are statistically significant.

## 3. Results

### 3.1. Comparison of General Data of the Two Groups

There was no statistically significant difference between the control group and the observation group in terms of gender, age, occupation, place of residence, smoking history, drinking history, underlying diseases, etiology, and causative factors (*P* > 0.05) (Table 1).

The article "Impact of Optimizing the Emergency Care Process on the Emergency Effect and Prognosis of Patients with Hepatic Encephalopathy" was published in 2022. Journal: Emerg Med Int.

### 3.2. Comparison of the Effect of First Aid between the Two Groups

The time spent on diagnosis, resuscitation, DTP, and DTT of patients in the observation group was much lower than that in the control group (*P* < 0.05). (Figure 1).

### 3.3. Comparison of Clinical Outcomes between the Two Groups

After resuscitation and follow-up treatment, 26 patients in the control group were discharged with cure, 4 patients were discharged with improvement, and 2 patients died of ineffective first aid, with a success rate of 93.72% (30/32). In the observation group, 29 patients were discharged with cure, 5 patients were discharged with improvement, and 0 patients died of ineffective first aid, with a success rate of 100% (34/34). The success rate of first aid in the observation group was higher than that in the control group, but the difference was not statistically significant (*P* > 0.05) (Figure 2).

### 3.4. Comparison of Nursing Quality between the Two Groups

The scores related to each quality of care, such as ambulance technique, humanistic care, resuscitation efficiency, and resuscitation effect, were significantly higher in the observation group than in the control group (*P* < 0.05) (Figure 3).

### 3.5. Comparison of Family Satisfaction between the Two Groups

After emergency care and after obtaining the consent of the family, the families of the patients in both groups were invited to evaluate the degree of satisfaction with clinical care based on the dimensions of the speed of emergency care, professionalism of the emergency nursing staff, and sense of responsibility for emergency care. In the control group, the percentages of very satisfied, basic satisfaction, and dissatisfaction with nursing care were 46.88%, 25.00%, and 28.13%, respectively, with a satisfaction rate of 71.88%. In the observation group, 76.47%, 17.65%, and 5.88% were very satisfied, basically satisfied, and dissatisfied with the nursing care, respectively, with a satisfaction rate of 94.12%. Statistical analysis of satisfaction between the two groups showed that the observation group was significantly higher than the control group (*P* < 0.05) (Table 2).

## 4. Discussion

HE is a syndrome of neuropsychiatric abnormalities of varying severity based on metabolic disorders caused by acute or chronic severe hepatic dysfunction of various etiologies or various portal vein-body circulation shunt abnormalities, mostly induced by upper gastrointestinal bleeding, constipation, infection, high-protein diet, and electrolyte disturbances [12–14]. The clinical manifestations of HE are diverse, manifesting only as reduced attention, memory, or abnormal brain electrophysiology in the early stages of the disease, and as the disease progresses, symptoms of neurological dysfunction such as drowsiness, delirium, or even coma may appear [15]. Studies [16, 17] have shown that HE can cause serious pathological changes related to cerebral edema, gastrointestinal bleeding, renal insufficiency, etc. If patients do not receive timely and effective treatment, it can cause sequelae of multisystem functional disruption and affect their normal life. At present, there is no specific clinical treatment for HE, and most of the treatment measures are comprehensive, while the factors affecting the prognosis of HE are treated as early as possible, but because the pathogenesis of HE is still unclear, there are few effective means of diagnosis and treatment, resulting in a very high mortality rate.

The article "Impact of Optimizing the Emergency Care Process on the Emergency Effect and Prognosis of Patients with Hepatic Encephalopathy" was published in 2022. Journal: Emerg Med Int.

Studies [18, 19] have shown that the traditional resuscitation care procedures are mainly focused on the rescue after the emergence of the problem, and the prognostic impact of the operations related to the assessment and prognosis of the disease, detailed management, and the interface of the resuscitation process is easily neglected, so there is a high risk of procedural confusion and delayed implementation of care measures in the rescue of HE patients, even if the health care workers are experienced and competent, which makes it difficult to ensure the effectiveness and orderliness of resuscitation. Optimizing the emergency care process means fully mobilizing the role of the nursing staff in the emergency department in the resuscitation procedure, when the emergency department receives the nursing staff to assess the patient's condition and immediately carry out life-saving measures as well as improve the success rate of emergency resuscitation [20]. The results of this study showed that the DTP, DTT, emergency time, and condition diagnosis time of the observation group were shorter than those of the control group, and the mortality rate was lower than that of the control group, suggesting that optimizing the emergency care process in the clinical treatment of HE patients can significantly reduce the adverse prognosis of patients, shorten the emergency time and condition diagnosis time, and relieve the clinical symptoms of patients. After optimizing the emergency care process, a standard emergency care process can reduce the unnecessary links, and the patient's condition can be assessed systematically, comprehensively, and in a timely manner to avoid delaying the emergency time due to multidisciplinary consultation, which can not only improve the success rate of resuscitation but also improve the resuscitation effect [21, 22].

The article "Impact of Optimizing the Emergency Care Process on the Emergency Effect and Prognosis of Patients with Hepatic Encephalopathy" was published in 2022. Journal: Emerg Med Int.

At the same time, close monitoring of changes in patients' vital signs and systemic reactions during resuscitation and observation of whether the operation method affects patients' physiology can fully reflect the humanistic care in resuscitation [23]. The results of this study showed that the quality of care scores in the observation group was significantly higher than those in the control group; this indicates that resuscitation of HE patients according to the optimized emergency care process can ensure the quality of care while ensuring the effectiveness of resuscitation. In addition, the results of this study also showed that the family members of the observation group were significantly more satisfied with the nursing care than the control group. The optimization of the emergency care process involved monthly nursing meetings, the formulation and implementation of solution measures in conjunction with the problems of emergency nursing staff in the process of HE emergency care, the regular implementation of skill training examinations for emergency nursing staff, and communication between nursing staff and patient's families to stabilize the patient's family emotions so that the patient's family could feel the care from the medical staff and thus receive good feedback.

In conclusion, the application of an optimized emergency care process in HE patients is effective, which can effectively improve the success rate of HE resuscitation, shorten the resuscitation time and diagnosis, enhance the resuscitation effect, and improve the quality of care, and is worthy of clinical promotion.

## Figures and Tables

**Figure 1:** Comparison of the effect of first aid between the two groups. Note. ▲ indicates *P* < 0.05 compared with the control group.

**Figure 2:** Comparison of clinical outcomes between the two groups.

**Figure 3:** Comparison of nursing quality between the two groups. Note. ▲ indicates *P* < 0.05 compared with the control group.

**Table 1:** Comparison of general data of the two groups.

Information		Control group (*n* = 32)	Observation group (*n* = 34)	*t* or *χ*^2^ value	*P* value
Gender (female, mean ± SD)		10 (31.25)	12 (35.29)	0.121	0.728
Age (years, mean ± SD)		50.25 ± 10.13	51.46 ± 9.77	0.494	0.623
Occupation (n, %)	Employee	4 (12.50)	5 (14.71)	2.040	0.844
	Worker	2 (6.25)	2 (5.88)		
	Farmer	1 (3.13)	2 (5.88)		
	Self-employed	0 (0.00)	1 (2.94)		
	Retired	15 (46.88)	17 (50.00)		
	Unemployed	10 (31.25)	7 (20.59)		
Geography (n, %)	Urban	24 (75.00)	28 (82.35)	0.533	0.465
	Rural	8 (25.00)	6 (17.65)		
Etiology (n, %)	Cirrhotic disease	26 (81.25)	27 (79.41)	0.035	0.851
	Noncirrhotic disease	6 (18.75)	7 (20.59)		
Causes (n, %)	Infection	15 (46.88)	18 (52.94)	0.243	0.622
	Upper gastrointestinal bleeding	12 (37.50)	11 (32.35)	0.192	0.661
	Electrolyte disturbances	13 (40.63)	16 (47.06)	0.277	0.599
	Diarrhea, constipation	4 (12.50)	5 (14.71)	0.068	0.794
	Others	2 (6.25)	4 (11.76)	0.607	0.436
Smoking history (n, %)		11 (34.38)	14 (41.18)	0.324	0.569
Alcohol consumption history (n, %)		12 (37.50)	14 (41.18)	0.093	0.760
Underlying disease (n, %)	Diabetes mellitus	4 (12.50)	6 (17.65)	0.138	0.933
	Coronary heart disease	1 (3.13)	1 (2.94)		
	Hypertension	4 (12.50)	7 (20.59)		

The article "Impact of Optimizing the Emergency Care Process on the Emergency Effect and Prognosis of Patients with Hepatic Encephalopathy" was published in 2022. Journal: Emerg Med Int.

**Table 2:** Comparison of family satisfaction between the two groups (n, %).

Group	Very satisfied	Basically satisfied	Unsatisfied	Satisfied
Control group (*n* = 32)	15 (46.88)	8 (25.00)	9 (28.13)	23 (71.88)
Observation group (*n* = 34)	26 (76.47)	6 (17.65)	2 (5.88)	32 (94.12)
*χ* ^2^ value	—	—	—	5.872
*P* value	—	—	—	0.015

## Data Availability

Raw data related to the results of this trial are available from the corresponding author.
